# Muscle Energy Technique plus Neurac Method in Stroke Patients with Hemiplegia Complicated by Diabetes Mellitus and Assessment of Quality of Life

**DOI:** 10.1155/2022/6318721

**Published:** 2022-05-09

**Authors:** Jingyan Wang, Shuang Wang, Hongmei Wu, Shuxin Dong, Baojun Zhang

**Affiliations:** Department of Rehabilitation Medicine, First Affiliated Hospital of Jiamusi University, Jiamusi, China

## Abstract

**Objective:**

To analyze the role of muscle energy technique (MET) plus Neurac method in stroke patients with hemiplegia complicated by diabetes mellitus and the impact on quality of life.

**Methods:**

From January 2021 to December 2021, 100 stroke patients with hemiplegia complicated by diabetes mellitus treated in our institution and assessed for eligibility were recruited and randomly assigned (1 : 3) via the random sampling method to either the conventional rehabilitation group or the experimental group. The patients in the experimental group were randomized (1 : 1 : 1) into either the MET group (receives MET), the Neurac group (receives Neurac), or the joint group (receives MET plus Neurac). The primary endpoint is the clinical efficacy, and the second endpoint is the quality of life.

**Results:**

The eligible patients had similar pretreatment Barthel index scores, Visual Analogue Scale (VAS) scores, Berg balance scale (BBS) scores, Tinetti scores, Fugl-Meyer scores, and quality of life (QoL) scores (*P* > 0.05). The treatment herein achieved significant improvements in Barthel index scores, VAS scores (2.71 ± 0.28), BBS scores, Tinetti scores, Fugl-Meyer scores, and QoL scores (99.67 ± 10.62), and MET plus Neurac method obtained the best results versus both the conventional rehabilitation and monotherapy of either MET or Neurac (*P* < 0.05).

**Conclusion:**

Neurac method plus MET improves the independent mobility of stroke patients with hemiplegia and diabetes, relieves pain, enhances balance and stability, mitigates limb dysfunction, and boosts patients' quality of life, so it is worthy of clinical application.

## 1. Introduction

Stroke is a group of acute diseases that include ischemic stroke and hemorrhagic stroke due to sudden rupture of blood vessels in the brain or failure of blood flow to the brain after vascular obstruction [1, 2]. Currently, functional impairment resulting in poor self-care abilities is associated with 70%-80% of stroke patients, such as limitation of motor function, sensory deficits, cognitive impairment, and speech and swallowing disorders, among which limited motor function severely compromises the daily life of hemiplegic patients [3, 4]. Moreover, the presence of knee hyperextension, knee hyperflexion, and inversion of the foot may lead to a failure of normal weight-bearing in the lower extremities in the support phase, which increases the patient's risk of falling. The close association of diabetes mellitus and cerebrovascular events constitutes an independent risk factor for stroke, and the comorbidity with diabetes mellitus may further aggravate the disease and cause a poor prognosis [5, 6]. Thus, an urgent need exists to explore effective rehabilitation treatment methods to improve the motor function and the quality of life of stroke patients with hemiplegia and diabetes mellitus. MET is a technique for musculoskeletal system disorders by applying isometric contraction, relaxation, and reciprocal inhibition to the targeted muscles. It relaxes tense muscles, activates relaxed muscles, and restores muscle length, tone, and stability to enhance the function of the musculoskeletal system and alleviate pain [7, 8]. In MET, patients are required to use their muscles to proactively and consciously fight against the resistance imposed by the therapist by using specific muscles to perform contraction, relaxation, and cross-inhibition to adjust muscle length and tone, increase muscle strength and stability, and restore the normal biomechanics of the joint, thereby achieving good therapeutic results [9–11]. The Neurac method is derived from sling exercise, where the patient receives rehabilitation using a sling system with the aid of the physical therapist, which allows reconstruction of normal movement patterns through high levels of neuromuscular stimulation. This approach has been applied in the treatment of long-term skeletal muscle disorders that cause pain or loss of function [12]. At present, the efficiency of the two treatment methods is marginally explored in treating patients with stroke hemiplegia and diabetes mellitus. Accordingly, this study was conducted to assess their efficacy in stroke patients with hemiplegia complicated by diabetes mellitus and the impact on quality of life, to further provide new ideas and directions in clinical practice.

## 2. Materials and Methods

### 2.1. Baseline Data

From January 2021 to December 2021, 100 stroke patients with hemiplegia complicated by diabetes mellitus treated in our institution and assessed for eligibility were recruited. They were concurrently randomly assigned via the random sampling method to either the conventional rehabilitation group (*n* = 25) or the experimental group (*n* = 75). The patients in the experimental group were randomized (1 : 1 : 1) into either the MET group (receives MET, *n* = 25), the Neurac group (receives Neurac, *n* = 25), or the joint group (receives MET plus Neurac, *n* = 25). All eligible patients showed comparable baseline characteristics (conventional rehabilitation group: 15 males and 10 females, aged 48-69 years, mean age of 57.45 ± 4.96 years, course of disease of 25-55 days, mean course of disease of 30.12 ± 4.27 days, 12 cases of cerebral infarction, and 13 cases of cerebral hemorrhage; MET group: 16 males and 9 females, aged 45-70 years, mean age of 58.30 ± 4.73 years, course of disease of 23-57 days, mean course of disease of 31.44 ± 4.38 days, 11 cases of cerebral infarction, and 14 cases of cerebral hemorrhage; Neurac group: 14 males and 11 females, aged 43-68 years, mean age of 56.98 ± 4.64 years, course of disease of 23-58 days, mean course of disease of 31.37 ± 4.50 days, 10 cases of cerebral infarction, and 15 cases of cerebral hemorrhage; and joint group: 17 males and 8 females, aged 43-70 years, mean age of 58.19 ± 4.55 years, course of disease of 22-56 days, mean course of disease of 30.72 ± 4.59 days, 16 cases of cerebral infarction, and 9 cases of cerebral hemorrhage (*P* > 0.05)). This protocol was approved by the ethics committee of the First Affiliated Hospital of Jiamusi University (JMUH39771).

### 2.2. Inclusion and Exclusion Criteria

Inclusion criteria are as follows: ① patients met the diagnostic criteria established for stroke in Chinese medicine and Western medicine (fasting blood sugar > 7.0 or two hours postprandial blood sugar > 11.1 mm/L) [13] and were confirmed by imaging CT or MRI for the first stroke with a duration of ≤3 months; ② aged between 18 and 79 years old, with normal heart rate, blood pressure, body temperature, and pulse; and ③ the enrolled patients had Glasgow Coma Scale scores of no less than 15 points, muscle strength of grade 2 or higher, and were able to cooperate actively. Patients and their families voluntarily participated in this experimental study and signed the informed consent form.

Exclusion criteria are as follows: ① patients with severe aphasia and cognitive dysfunction; ② with a previous history of psychiatric disorders; and ③ with severe infections, heart failure, tumors, asthma, and other serious complications or hepatic dysfunction or renal dysfunction.

### 2.3. Methods

The conventional rehabilitation group adopted conventional rehabilitation training. Patients received conventional diabetes treatment, regular blood glucose monitoring, medication as prescribed by the doctor, and dietary guidance. The rehabilitation training included active and passive activities of the hemiplegic side of the limb, turning and movement training, early healthy limb position placement, muscle strength training, balance training, occupational therapy, walking training, traditional rehabilitation therapy, and physiotherapy, 40 min/time, 1 time/d, 5d/week, for a total of 4 weeks.

Patients in the MET group were given MET on top of conventional treatment. (1) Respiratory training (to help ease the overexcited sympathetic nerves): in a supine position, the patient was instructed to bend the hips and knees and place the feet on the Bobath ball and breathe with a relaxed abdomen. The therapist placed both hands on the patient's abdomen and instructed the patient to do a slow “yawn-like” exhalation, and the therapist slowly pressed both hands onto the abdomen to promote diaphragmatic uplift. Patients held their breath for 5-10 s at the end of exhalation, 10 sets/time. (2) Tension-reducing isometric contraction-relaxation technique for pectoralis major and pectoralis minor: the patient lied in a supine position with the head turned to the opposite side of the training side and the shoulder joint abducted at 90° hanging out of the bed. The therapist pressed the patient's pectoralis major with one hand and held the patient's elbow with the other, rotated the shoulder externally and pressed down to a point where the patient could feel resistance without pain and instructed the patient to use 20% of maximum contraction against the resistance and relax after holding for 5-10 s. The therapist then continued to stretch to the next new resistance point and repeated 3-5 times. The middle and lower part of the muscle strength enhancement training was used for the rhomboid muscles and trapezius. The patient was seated with the shoulder abducted at 90° on the table. The therapist instructed the patient to contract the scapula inwards and placed the hand on the medial side of the scapula to apply resistance outward, 20 pieces/set, 3-5 sets/time. Shoulder joint hold-relaxation technique: with the patient in a seated position, the therapist assisted the patient to flex the shoulder joint forward to the point where the patient could feel the resistance without pain and instructed the patient to remain still. The therapist appropriately applied resistance at the distal end of the upper extremity according to the actual condition. The resistance should be reduced immediately in the case of compensatory movements such as shrugging. The patient maintained for 5-10 s and then slowly relaxed, after which the therapist stretched the shoulder to a next resistance point for training and repeated 3-5 times. (3) Treatment of the elbow joint: biceps isometric contraction-relaxation training: with the patient in a supine position and the forearm rotated back in a neutral shoulder position, the therapist slowly stretched the patient's elbow to a point of resistance without pain and instructed the patient to use 20% of the maximum contraction force against it to achieve an isometric contraction, hold for 5-10 s, and then relax, after which the stretch was continued to the next new point of resistance and repeated 3-5 times. Triceps centrifugal MET training: the therapist assisted the patient to straighten the elbow joint to the maximum angle, held the patient's wrist joint, and applied resistance in the direction of elbow flexion, and the patient kept passively flexing the elbow joint to the maximum under confrontation, 20 pieces/set, 3-5 sets/time. (4) Wrist training: the therapist dorsally stretched the patient's wrist to a point of resistance without pain and instructed the patient to use 20% of the maximum contraction force against it to achieve isometric contraction, hold for 5-10 s, and then relax, and the therapist then dorsally stretched the wrist to the next new point of resistance and repeated 3-5 times. Centrifugal training of wrist extensors: the therapist instructed the patient to dorsally extend the wrist joint to the maximum angle, immobilized the wrist joint in the palmar flexion direction, and applied a constant resistance, and the patient maintained passive palmar flexion under confrontation to the maximum, 20 pieces/set, 3-5 sets/time.

The Neurac group used the Neurac method for training. (1) Supine pelvic lifting: using an elastic cord attached to a wide sling placed at the pelvis, the knee joint was kept straight by pressing down on the rigid knee sling so that the body would not rotate and flex laterally, which can increase lower limb muscle strength and impedance through repetitive training. The adjustment of the length of the elastic cord helps to reduce the weight-bearing to accommodate the patient's physical condition [14]. (2) Lateral recumbent hip abduction: the therapist instructed the patient to lift the healthy leg, extend the hip, and use straightening of the affected leg and downward pressure on the rigid narrow sling to lift the body so that the seventh thoracic vertebra and the inner ankle of the affected limb could be on the same level. The patient was only required to maintain a normal physiological curvature without side-bending and rotation. (3) Lateral recumbent hip inversion: with the patient's head resting on a pillow or arm and the other arm placed at the forehead, a nonelastic cord was placed near the knee joint of the upper leg at a height such that the lower edge of the knee joint of the upper leg was slightly above shoulder level, and the elastic cord was placed at the pelvis with the central point of each sling suspended. The spinal curvature should be kept within a normal range during training. The lower leg was lifted off the bed and pressed down to raise the pelvis, and the body was to be kept straight with normal spinal curvature and the lower hip in a posterior extension position without lateral flexion or rotation of the body [15]. (4) Neutral lumbar spine position in a supine position: the length of the rigid cord was adjusted to allow hip flexion > 30°, and the treatment bed was lowered to bring the pelvis off the bed. Adjustment of the elastic cord at the pelvis enables the therapist to adjust the curvature of the lumbar spine using less force. For patients with upper extremity dysfunction, the patient was instructed to kneel and then straighten the arms until the shoulder joint was flexed at 90° and then performed a push-up. This is followed by supine shoulder abduction: the hand strap was placed on both elbows above shoulder height, with the split sling applied to the head and the wide sling applied under the upper back, and the pelvis was to offload the weight. The patient then extended the knees and hips, lifted the body off the treatment table, and abducted the straightened arm 180°.

The patients in the joint group were treated with MET plus Neurac method, and the specific treatment methods were the same as those in the MET and Neurac groups. All four groups of patients underwent 4 weeks of training and were followed up by telephone 1 month after treatment.

### 2.4. Outcomes

(1) The Barthel (BI) index scale was used to assess patients' quality of daily living before, 2 weeks after, and 4 weeks after treatment, including items such as dressing, body transfer, walking, and bowel and urinary control. The total score of each item was 100 points. 100 points mean independent daily living; 61-99 points are mild impairment of daily life and occasionally require assistance; 41-60 points are moderate dependence and mostly require assistance; ≦40 points mean severe dependence and require full-time care. (2) Visual Analogue Scale (VAS): pain was divided into 0-10 levels on this sliding scale, with 0 points indicating no pain and 10 points indicating unbearable pain. A personal check was made on a piece of paper marked with 10 intervals with 0 for no pain and 10 for maximum pain. This test tool has a test-retest reliability. (3) Berg balance scale (BBS): the BBS was used to assess the balance function of hemiplegic patients: the sum of the scores was 56 points, and the higher the scores, the better the balance ability of the stroke patients. A sum of all scores less than 40 points indicates a risk of falling. Fourteen items are assessed to determine the patients' ability to maintain balance through sitting, standing, and postural changes, and about 20  minutes is taken. If the items cannot be performed at minimum, 0 points are given, and for completely independent, the maximum of 4 points is noted. (4) Tinetti gait assessment: gait assessment items include the starting step, lifting height, step length, gait symmetry, stride continuity, walking path, trunk stability, and step width. The full score is 12 points, where the walking path and trunk stability are scored on three levels of 0, 1, and 2 points, and the other items are scored on two levels of 0 points and 1 point. (5) The Fugl-Meyer scale was applied to assess the motor function of the lower extremities, and the main items include neuroreflex activity, common flexor movement, common extensor movement, joint common movement, detachment movement, and coordination/speed, with a full score of 34 points: (I) unsupported sitting: 0 points: unable to maintain the sitting position; 1 point: able to sit, but less than 5 minutes; and 2 points: able to sit for more than 5 minutes; (II) unaffected wing spread response: 0 points: no shoulder abduction or elbow joint extension, 1 point: weakened response, and 2 points: the response is normal; (III) wing-spreading response on the affected side: the score is the same as that of item (II); (IV) standing under support: 0 points: unable to stand, 1 point: can stand under the maximum support of others, and 2 points: able to stand for 1 minute with a little support from others; (V) standing without support: 0 points: unable to stand, 1 point: unable to stand for more than 1 minute, and 2 points: able to balance standing for more than 1 minute; (VI) standing on the healthy side: 0 points: unable to maintain 12 seconds, 1 point: able to balance standing for 49 seconds, and 2 points: able to balance standing for more than 10 seconds; (VII) standing on the affected side: the score is the same as item (VI). (6) The WHO/Q0L-26 World Health Organization Quality of Life Measurements Short Form (WHOQOL-BREF) was used to assess patients' quality of life, which includes 5 domains (physical, psychological, social, environmental, and integrated) and 26 items with a total score of 130 points. The higher the score, the better the quality of life. All questions are rated on a 5-point Likert scale, and the item is scored between 1 and 5. Raw scores in each domain were changed to a 4–20 score based on the guideline. All domain scores were linearly changed such that they varied from 0 to 100 with “100” demonstrating the highest possible QoL.

### 2.5. Statistical Analysis

SPSS 20.0 was used for data analyses, and GraphPad Prism 7 (GraphPad Software, San Diego, USA) was used to visualize the data into corresponding images. The count data were expressed as *n* (%) and processed using the *χ*^2^ test, and the measurement data were expressed as ($\overset{®}{x}\pm s$) and processed using the *t*-test. Differences were considered statistically significant at *P* < 0.05.

## 3. Results

### 3.1. Barthel Index Scores

The pretreatment Barthel index scores were similar among all eligible patients (*P* > 0.05). All treatment methods adopted in the present study showed significant enhancement in the Barthel index scores, with the best results observed in the joint group (*P* < 0.05) (Table 1).

### 3.2. Comparison of VAS Scores

No significant differences were obtained in VAS scores among the four groups of patients (*P* > 0.05). After treatment, all patients obtained markedly decreased VAS scores, and those receiving the combined therapy had the lowest scores versus those of other groups (*P* < 0.05) (Table 2).

### 3.3. BBS Scores

The pretreatment BBS scores were similar in all eligible patients (*P* > 0.05). After treatment, a remarkable increase in the BBS scores in all four groups was observed, with the best results achieved by the joint group (*P* < 0.05) (Figure 1).

### 3.4. Tinetti Scores

Before treatment, the four groups presented similar Tinetti scores (*P* > 0.05). After treatment, the joint group showed significantly higher Tinetti scores versus the other treatment methods (*P* < 0.05) (Figure 2).

### 3.5. Fugl-Meyer Scores

Before treatment, no significant differences were obtained in the Fugl-Meyer scores among the four groups (*P* > 0.05). After treatment, the Fugl-Meyer scores of the four groups were increased significantly, with the highest results obtained in the joint group (*P* < 0.05) (Table 3).

### 3.6. QoL Scores

The pretreatment QoL scores were similar among the four groups of patients (*P* > 0.05). After treatment, MET plus Neurac achieved more significant improvements in the quality of life versus the other groups (*P* < 0.05) (Table 4).

## 4. Discussion

The loss of control of higher centers over lower centers after the onset of stroke leads to sensory, motor, speech, swallowing, and cognitive dysfunction, and the disease has a high prevalence, which seriously jeopardizes patients' health and life safety [16]. Most patients are prone to hemiparesis, aphasia, and decreased limb function, where hemiparesis occurs due to loss and decrease in coordination between various muscle groups after stroke, leading to impaired motor and static balance and trunk control [17, 18]. Comorbid diabetes mellitus in stroke patients aggravates brain tissue damage and increases the disability rate. Research has shown [19] that hyperglycemia causes decreased erythrocyte activity in the body and damage to vascular endothelial tissue, promotes the development of atherosclerosis and thrombosis, and aggravates the degree of cerebral infarction and injury. Moreover, hypoglycemia compromises the neurological and cardiovascular systems of stroke patients, resulting in cognitive dysfunction [20]. Therefore, effective rehabilitation training plays an important role in the recovery of limb functions and improving the quality of life. Conventional rehabilitation training applied in stroke patients with hemiplegia combined with diabetes can improve the limb motor function of patients but fails to achieve the desired effectiveness [21]. MET promotes blood supply to muscle fibers through activation of target muscles, which contributes to the reconstruction and strengthening of tissue fibers, stretching contracted muscle fibers, enhancing muscle strength, increasing the range of motion of joints, and promoting the uniform distribution of external forces to the individual muscles of the restored stable muscle groups. In addition, the active contraction and diastole of the muscles allow the soft tissues around the joints to form spirals or inspirals, which accelerates the movement of the body's deep cells and body fluids, facilitating the elimination of stagnant material and speeding up the rate of tissue reoxidation and removal of metabolites [22]. The Neurac method is a neuromuscular functional training technique used to treat long-term skeletal muscle disorders and is derived from sling therapy, where the patient is gradually rehabilitated through a sling system and the assistance of a physical therapist. It is used to reestablish normal movement patterns through high levels of neuromuscular stimulation.

In the present study, all eligible patients obtained significantly elevated Barthel index scores, and MET plus Neurac presented the best results versus other treatment methods, indicating that patients had significant improvement in limb function through rehabilitation training and were able to perform certain activities of daily living independently and that the combination of MET and Neurac potentiates the treatment effectiveness. The increased VAS scores after treatment and the highest scores observed in the joint group suggested that the combined treatment better alleviated the pain during rehabilitation training. A study by Wolf et al. [23] used the MET in rehabilitation training for patients after anterior cruciate ligament reconstruction, and the scoring of knee pain found that the inclusion of the MET in rehabilitation training reduced pain and facilitated the functional rehabilitation of patients. The significantly higher elevation of BBS scores and Tinetti scores of the joint group after treatment indicates that the combination treatment can improve the patient's balance, increase the stability of walking, and reduce the risk of falling. MET enhances the balance of the muscle groups around the joint by lengthening the tense and shortened muscle groups and strengthening the relaxed and elongated muscle groups, to restore the normal biomechanics of the joint. The Neurac method assists patients' active movement with the aid of sling movement system, using open chain and closed chain movements for training, which can more effectively improve the coordinated contraction of muscle groups, enhance the weak links of trunk stabilizing muscle groups and power muscle groups, strengthen patients' control of the trunk, and reinforce the balance control and stability state. Here, the combination of MET and Neurac method obtained significantly higher Fugl-Meyer versus conventional rehabilitation and monotherapy of either MET or Neurac, which was similar to the findings of SAMUEL [24] et al., suggesting that MET combined with the Neurac method could improve the dysfunction of patients' lower limbs, activate nerves and muscles, and restore muscle strength, allowing patients to reestablish normal movement patterns. In addition, the superior quality of life of patients receiving joint treatment in the present indicates better quality of life benefits of joint treatment.

To sum up, Neurac method plus MET improves the independent mobility of stroke patients with hemiplegia and diabetes, relieves pain, enhances balance and stability, mitigates limb dysfunction, and boosts patients' quality of life, so it is worthy of clinical application.

## Figures and Tables

**Figure 1:** Comparison of BBS scores. Note: The abscissa indicates pretreatment, 2 weeks of treatment, and 4 weeks of treatment; the ordinate indicates BBS score, points. The BBS scores of the conventional rehabilitation group before treatment, 2 weeks of treatment, and 4 weeks of treatment were 28.17 ± 2.55, 37.69 ± 2.12, and 45.30 ± 1.83, respectively. The BBS scores before treatment, at 2 weeks of treatment, and at 4 weeks of treatment in the MET group were 27.94 ± 2.48, 42.37 ± 2.26, and 48.65 ± 3.01, respectively. The BBS scores before treatment, at 2 weeks of treatment, and at 4 weeks of treatment in the Neurac group were 28.11 ± 2.35, 43.18 ± 2.42, and 49.04 ± 2.81, respectively. The BBS scores before, 2 weeks, and 4 weeks of treatment in the joint group were 27.61 ± 2.47, 48.16 ± 3.20, and 53.17 ± 1.87, respectively. ∗ and # indicate significant differences in the BBS scores between the conventional rehabilitation group and the joint group after 2 weeks of treatment and 4 weeks of treatment (*t* = 13.638, 15.039, *P* < 0.001). ∗∗ and ## indicate significant differences in the BBS scores between the MET group and the joint group after 2 weeks of treatment and 4 weeks of treatment (*t* = 7.390, 6.377, *P* < 0.001). ∗∗∗ and ### indicate significant differences in the BBS scores between the Neurac group and the joint group after 2 weeks of treatment and 4 weeks of treatment (*t* = 6.206, 6.118, *P* < 0.001).

**Figure 2:** Comparison of Tinetti scores. Note: The abscissa indicates pretreatment, 2 weeks of treatment, and 4 weeks of treatment; the ordinate indicates Tinetti score, points. The Tinetti scores of the conventional rehabilitation group before, 2 weeks, and 4 weeks of treatment were 3.27 ± 0.35, 5.52 ± 0.41, and 7.38 ± 0.51, respectively. The Tinetti scores before treatment, at 2 weeks of treatment, and at 4 weeks of treatment in the MET group were 3.10 ± 0.29, 7.37 ± 0.63, and 8.32 ± 0.74, respectively. The Tinetti scores before treatment, at 2 weeks of treatment, and at 4 weeks of treatment in the Neurac group were 3.08 ± 0.30, 7.59 ± 0.65, and 8.46 ± 0.78, respectively. The Tinetti scores before, at 2 weeks, and at 4 weeks of treatment in the combined group were 3.13 ± 0.25, 8.72 ± 0.44, and 10.37 ± 0.81, respectively. ∗ and # indicate significant difference in the Tinetti scores between the conventional rehabilitation group and the joint group after 2 weeks of treatment and 4 weeks of treatment (*t* = 26.604, 15.619, *P* < 0.001). ∗∗ and ## indicate significant differences in the Tinetti scores between the MET group and the joint group after 2 weeks of treatment and 4 weeks of treatment (*t* = 8.784, 9.343, *P* < 0.001). ∗∗∗ and ### indicate significant differences in Tinetti scores between the Neurac group and the joint group after 2 weeks and 4 weeks of treatment (*t* = 7.198, 8.493, *P* < 0.001).

**Table 1:** Comparison of Barthel index scores.

Groups	Before treatment	2 weeks of treatment	4 weeks of treatment
Conventional rehabilitation group	35.59 ± 4.16	40.37 ± 5.44	56.91 ± 7.33
MET group	33.91 ± 5.10	52.41 ± 6.56^∗^^#^	62.43 ± 8.10^∗^^#^
Neurac group	34.72 ± 4.96	53.72 ± 6.83^∗^^#^	63.59 ± 8.26^∗^^#^
Joint group	35.46 ± 4.24	60.59 ± 8.17^∗^	80.28 ± 9.47^∗^

∗ indicates *P* < 0.05 versus conventional rehabilitation group within the same time period; # indicates *P* < 0.05 versus the joint group.

**Table 2:** Comparison of VAS scores.

Groups	Before treatment	2 weeks of treatment	4 weeks of treatment
Conventional rehabilitation group	8.36 ± 0.75	6.28 ± 1.05	5.37 ± 0.69
MET group	8.29 ± 0.81	5.46 ± 0.78^∗^^#^	4.41 ± 0.42^∗^^#^
Neurac group	8.59 ± 0.94	5.40 ± 0.728^∗^^#^	4.39 ± 0.50^∗^^#^
Joint group	8.74 ± 1.02	4.12 ± 0.528^∗^	2.71 ± 0.28^∗^

∗ indicates *P* < 0.05 versus conventional rehabilitation group within the same time period; # indicates *P* < 0.05 versus the joint group.

**Table 3:** Comparison of Fugl-Meyer scores.

Groups	Before treatment	2 weeks of treatment	4 weeks of treatment
Conventional rehabilitation	14.69 ± 3.12	18.01 ± 4.25	20.54 ± 4.33
MET group	15.28 ± 3.04	20.75 ± 3.67^∗^^#^	23.44 ± 4.19^∗^^#^
Neurac group	14.74 ± 2.98	20.66 ± 2.58^∗^^#^	24.02 ± 3.95^∗^^#^
Joint group	15.21 ± 2.71	23.34 ± 2.16^∗^	29.16 ± 3.08^∗^

∗ indicates *P* < 0.05 versus conventional rehabilitation group within the same time period; # indicates *P* < 0.05 versus the joint group.

**Table 4:** Comparison of QoL scores.

Groups	Before treatment	2 weeks of treatment	4 weeks of treatment
Conventional rehabilitation group	41.27 ± 5.13	56.71 ± 7.28	75.42 ± 8.26
MET group	42.54 ± 5.29	65.83 ± 8.10^∗^^#^	86.19 ± 10.22^∗^^#^
Neurac group	41.38 ± 5.07	67.34 ± 8.50^∗^^#^	87.37 ± 10.15^∗^^#^
Joint group	43.15 ± 5.12	74.60 ± 9.25^∗^	99.67 ± 10.62^∗^

∗ indicates *P* < 0.05 versus conventional rehabilitation group within the same time period; # indicates *P* < 0.05 versus the joint group.

## Data Availability

The datasets used during the present study are available from the corresponding author upon reasonable request.
